# Nursing Education of Lateral Oblique Complications of Neurosurgery under Microscope

This article has been retracted.

**DOI:** 10.1155/2022/2158181

**Published:** 2022-08-05

**Authors:** Kecui Hu

**Affiliations:** School of Nursing, Anhui University of Chinese Medicine, Hefei, Anhui 230012, China

## Abstract

In order to solve the problem of nursing education of lateral oblique complications, a nursing education solution of lateral oblique complications of neurosurgery under the microscope was proposed. The method used subjective evaluation and objective evaluation to systematically evaluate the basic training module. In subjective evaluation, the authenticity score of surgical simulator was 3.65 ± 0.01, the realism score of surgical instruments was 3.81 ± 0.01, the realism score of tactile sense was 3.75 ± 0.01, the operating environment score was 3.60 ± 0.01, and the overall effect score was 3.63 ± 0.01. The difficulty score of the whole training was 3.15 ± 0.01. In the aspect of objective evaluation, the entropy method was used to process the data of training track, training angle, training time, trigger times, success times, failure times, and other indicators of 24 trainers collected, and the experiment verified the nursing education of lateral oblique complications of neurosurgery under the microscope.

## 1. Introduction

As one of the most technically demanding medical specialties, neurosurgery requires neurosurgeons not only to have a high level of theoretical knowledge but also to have high operational skills, in order to ensure the reduction of any unnecessary mistakes, because any mistakes will lead to serious consequences, so simulation surgery has become a daily training for every neurosurgeon to maintain their surgical skills, as shown in Figure 1. In modern times, simulation plays an extremely important role in both medical and nonmedical fields, especially in fields with high risk and high cost, including the training of military personnel, pilots, car drivers, and nuclear power plant operators. Through simulation, trainers can study and experiment with process interactions with different processes, consider various processes, monitor the impact of ideas on models and methods, perform, and select the best ideas. In medicine, simulated surgery is generally divided into physical simulation and virtual simulation. Physical simulations typically include cadaver models, live animal models, and artificial limb simulation models. Cadaver model and live animal model are the best training methods for surgeons to practice their surgical skills, but they have some problems such as lack of cadaver source and ethics. Prosthesis simulation is an alternative scheme, which can achieve 1 : 1 reduction through 3D printing. However, due to the limitation of materials, this scheme has low repeatability and cannot improve the real feeling of surgeons. Virtual simulation includes virtual reality, augmented reality, and mixed reality. Combined with the real operation environment, real-time tactile feedback can improve the immersion of training physicians, achieve the purpose of training physicians spatial sense, and improve surgical skills, which is a very promising training method at present.

## 2. Literature Review

Yan et al. said that the 2019 China Cancer Report released by the China Cancer Center indicated that about 10,000 people are diagnosed with cancer every day, an average of seven people every minute. The report pointed out that the most important treatment for cancer is surgery, so the training of surgical skills for surgeons has become particularly important [1]. Swiatek et al. said that with the rapid expansion of the enrollment of medical colleges in China, the difficulty in obtaining cadavers, the unguaranteed surgical training, the low efficiency, and high cost of the training of surgeons would greatly prolong the training cycle of a surgeon [2]. Krych et al. said that neurosurgery includes craniocerebral surgery, spinal neurosurgery, spinal neurosurgery, and peripheral neurosurgery. Craniocerebral surgery and spinal neurosurgery are the most important components of neurosurgery and also the two most studied directions outside China [3]. Martins et al. say that with the development of science and technology, the concept of minimally invasive surgery has permeated the whole process of neurosurgery and treatment. Not only can patients undergo painless neurosurgery, but with the development of visualization techniques such as magnetic resonance imaging (MRI), computed tomography (CT), and neuroendoscopy. Diagnosis and treatment of neurological diseases have become more reliable [4]. Tamborska et al. stated that the Neurosurgical Navigation System (NNS) concept originated in the 1990s [5]. Ivanov et al. stated that NSS uses a high-performance computer to closely correlate patient preoperative image data (MRI and CT) with the actual location of intraoperative lesions. Surgeons can display three-dimensional (3D) images of surgical sites and instruments in real time through a monitoring screen [6]. Aibar-Duran et al. said that preoperative imaging often fails to provide accurate guidance to the surgeon due to changes in the patient's position or surgical environment [7]. Therefore, intraoperative imaging technology has attracted more and more attention, such as intraoperative MRI, intraoperative three-dimensional ultrasound, intraoperative CT, and other imaging technology 1. Agrawal et al. said that surgeons can fuse intraoperative images with preoperative planning images or omit preoperative images to simplify the intraoperative imaging process of image-guided neurosurgery work and provide more auxiliary information [8]. Andreev et al. said that the development of neurosurgery depends on advances in existing surgical techniques [9]. According to Febns et al., the results of computed tomography and magnetic resonance imaging have ushered in a new era in neurosurgery, with medical applications including surgical microscopy, ventricular endoscopy, intraoperative navigation, and multidirectional clinical trials. The idea of minimally invasive surgery has flooded [10]. However, current methods only use two test models, which is also a limitation for most new surgeons. VR was first used in medicine in the early 1990s to view difficult medical records during surgery and plan preoperative procedures. For 3D reconstruction, VR is considered one of the most promising surgical plans.

## 3. Methods

It indicates that the algorithm is a classical swarm algorithm. It is one of the partitioning process. The *k*-word algorithm uses *k* as a measure and divides *n* models into *k* groups. The goal is to make the samples within the cluster have high similarity, while the similarity between samples belonging to different clusters is low. The algorithm tries to find *k* partitions that reduce the squared error value, usually ending up in a local optimum. The *k*-language algorithm uses distance as a measure of similarity, that is, the closer the distance between two models, the greater the probability [11]. The algorithm considers that clusters are composed of samples that are close to each other, but samples belonging to different clusters are far apart, so compact and independent clusters can be obtained. *k* is assuming that there are *n* models in the configuration file, and each model has the characteristics of *P*; then, each model can be used as the following vector, as shown in the following formula:

(1) $$\begin{array}{c} X_{i}=\left(X_{1i},X_{2i},\cdots ,X_{\rho i}\right),i=1,2,3,\cdots ,n. \end{array}$$

*k* samples were selected as the initial clustering centers, and the following vectors of each clustering center are shown in the following formula:

(2) $$\begin{array}{c} Z_{\text{i}}=\left(z_{1j},z_{2j},\cdots ,z_{pj}\right),j=1,2,3,\cdots ,k. \end{array}$$

The calculation method usually uses the error sum of squares criterion function as a function of the group. The error sum of squares criterion function is defined by the following equation:

(3) $$\begin{array}{c} J_{c}=\overset{k}{\underset{j=1}{\sum }}\overset{n_{j}}{\underset{i=1}{\sum }}{\left\|x_{i}-m_{j}\right\|}^{2}, \end{array}$$

where *k* is the number of clustering to be formed, *η*_*j*_ is the number of samples in the *j*-th class, *m*_*j*_ is the mean value of class *J* samples and represents the center of gravity of this type of data set, as shown in the following formula:

(4) $$\begin{array}{c} m_{j}=\frac{1}{n}\overset{nj}{\underset{j=1}{\sum }}x_{j},j=1,2,\cdots ,k. \end{array}$$

The method of iterative updating is adopted: in each iteration, *k* clusters are formed according to the sample points around *k* cluster centers, and the centroid of each cluster obtained by recalculation (namely, the average value of all points in the cluster, namely, the set center) will be used as the reference point of the next iteration [12, 13]. The reference points selected iteratively are closer and closer to the real center of mass of the cluster, so the objective function is smaller and smaller, and the clustering effect is better and better [14]. First, select *k* points as the starting point according to the understanding of *k*, and then, calculate the distance from each model to the center point. Center the model where it is closest to it and adjust the position of the new group. If there is no change in the clustering center of two adjacent iterations, it indicates that the sample adjustment is over, the li number *J*_*c*_ of the clustering criterion has converged, and the algorithm is over.

Set the sample set size *n*, the number of clusters *k*, and the convergence criterion *ε*, let the number of iterations mark/ = *I*, and select *k* initial focal points *z*(*j*)(/) from the sample set, *j* = 1, 2 ⋯ *k*. The location *D*(*X*, *Z*, (/)), *i* = 1, 2.⋯ of each sample object from the cluster center was calculated, *j* = 1, 2 ⋯ *k* as shown in the following formula:

(5) $$\begin{array}{c} D\left(X_{i},Z\left(/\right)\right)=\min\left\{D\left(X_{i}\right.,Z\left(/\right)\right\},j=1,2,3,\cdots ,n. \end{array}$$

The standard function *J*_*c*_ of calculation error is shown in the following formula:

(6) $$\begin{array}{c} J_{c}\left(/\right)=\overset{k}{\underset{j=1}{\sum }}\overset{n_{i}}{\underset{m=1}{\sum }}{\left\|X_{m}^{\left(j\right)}-Z\left(/\right)\right\|}^{2}. \end{array}$$

AP algorithm is a new unsupervised clustering algorithm developed by Sc IENCC in 2007. The algorithm is a clustering algorithm based on data transfer between nodes. The goal of the job is to find the slope at the best position in the group such that the result for each data point is similar to the content of the group. The algorithm is fast and effective and has good application results in face image clustering, gene recognition, handwriting character recognition, and optimal air route planning. In the AP algorithm, two data types, responsible and available, are usually exchanged, where *r*(*i*, *k*) represents the number sent from point *i* to candidate group *k*, considering whether point *k* corresponds to the midpoint of point *i*. *A*(*i*, *k*) represents the number sent to me by candidate group *k*, considering how I choose *k* as its midpoint [15]. In fact, the process of AP algorithm iteration is to constantly update the attractiveness and belonging values of each data point and finally generate *M* cluster center points and then allocate the remaining data points to the corresponding cluster according to the similarity. The relationship between attractiveness and belonging is shown in Figure 2.

The core steps of AP clustering algorithm are the iterative updating of *r*(*i*, *k*) and *a*(*i*, *k*), and the updating formulas are shown as follows:

(7) $$\begin{array}{c} r\left(i,k\right)=s\left(i,k-\underset{j\neq k}{\max}\left\{a\left(i,j\right)+s\left(i,j\right)\right\}\right., \end{array}$$

(8) $$\begin{array}{c} a\left(i,k\right)=\min\left\{0,r\left(k,k\right)+\underset{j\neq i,j\neq k}{\sum }\max\left\{0,r\left(k,k\right)\right\}\right\},i\neq k. \end{array}$$

As shown in the following formula,

(9) $$\begin{array}{c} a\left(i,k\right)=\underset{j\neq k}{\sum }\max\left\{0,r\left(j,k\right)\right\}. \end{array}$$

During the entire iterative process of the algorithm, the *r*(*i*, *k*) and *a*(*i*, *k*) information values of each sample point are constantly updated by the algorithm until the convergence of the algorithm is completed. Thus, *k* high-quality exemplar can be generated, and then, the nonclustering centered exemplar. Data points are allocated to the corresponding cluster. Damping factor lam ∈ [0.5, 1] is introduced to avoid oscillation. Increasing dayani factor can effectively eliminate the oscillation and make the algorithm converge. lam = 0.9 can be obtained, as shown in the following formula:

(10) $$\begin{array}{c} r^{\left(t\right)}\left(i,k\right)=\left(1-\text{lam}\right)*\left[s\left(i,k\right)-\underset{j\neq k}{\max}\left\{a^{t-1}\left(i,j\right)+s\left(i,j\right)\right\}+\text{lam}*r^{\left(t-1\right)}\left(i,k\right)\right]. \end{array}$$

Means algorithm is widely used because of its simple theory and fast calculation speed. However, it also has many defects: the number of clustering in *k*-means algorithm needs to be given in advance. The clustering result depends on the reasonable choice of user parameters, but the selection of the number of clustering is very difficult to estimate, especially when we do not know the given data distribution form, so it is impossible to determine how many classes the data set should be divided into. The algorithm has great dependence on the selection of initial value. Different initial values often lead to different results, which leads to poor stability of the algorithm [16]. The *k*-means algorithm needs to update the distribution model regularly and continuously count new sites after modification. Therefore, when the data cost is very large, the time cost of the algorithm is very large. And the algorithm is sensitive to noise and outliers. In the face of the original data with complex human quantity and errors (action: operation of fire failure data), we first consider how to convert the original data into data in accordance with the requirements of mathematical analysis methods. The nursing bed movement history in the system of “multi-functional nursing and physiological parameters remote monitoring device” is the source data object of this paper. This data sheet includes six attributes: control mode (manual, voice, and timing control), action type, action time, action value, operation result, fault analysis, and remarks. Due to inevitable objective reasons, there are errors and omissions in the data, and the quality of the data will directly affect the clustering algorithm results, so it is necessary to preprocess the source data [17]. Nonparametric rank-sum test analysis showed that patients' satisfaction with nursing work in the intervention group was significantly better than that in the control group, and the difference between the two groups was statistically significant (*Z* = 3.479, *P* < 0.05), as shown in Table 1 and Figure 3.

## 4. Experiment and Analysis

The overall framework of the nursing bed experimental platform is shown in Figure 4.

The main control computer as a human-computer interaction interface and user input control signal platform, care bed motor control drive system to complete the analysis of control signal, and drive the corresponding control bed parts of the motor [18, 19]. The nursing bed should meet the various necessary positions and postures which are conducive to the nursing person's rehabilitation and self-care. For example, in order to prevent bedsores and a series of complications caused by poor blood flow due to a long time in bed, nursing bed can realize the bed surface left and right side turn over action. To speed up the healing of a patient's injured leg, the nursing bed offers leg lifts and more. The nursing bed has 12 single movements in total, and all single movements of the nursing bed are shown in Table 2 below.

They are left turn up, left turn down, right turn up, right turn down, back up, back down, leg up, leg down, head of the bed up, head of the bed down, bed end up, and bed end down. There are also two combined movements: bed rise and bed fall, which are made by the head and tail of the bed in coordination [20]. If bed body rises, namely, the head of a bed and bed end rise at the same time, bed body drops, namely, the head of a bed and bed end drop at the same time, because this nurses a bed to share 14 action types. The nursing bed consists of a number of independent institutions in mechanical structure, each corresponding to more than one degree of freedom. Under the unified and coordinated control of the control system, these institutions form a multichain system, through the cooperative movement of each bed panel, so that the nursing bed completes a specific posture [21]. Therefore, the design and implementation of the control system is one of the most important parts of the whole nursing bed. In order to make the control system realize intelligent control of nursing bed and timely understand the current working state of nursing bed, the necessary number of position sensors is installed on the nursing bed body. By detecting the data transmitted back through the sensor, the control system can understand the motion state of each bed panel in real time, to avoid the mutual interference of different institutions or the overimpact of the linear motor and other unnecessary damage to the bed and the user. Nursing bed movement control system adopts the control mode of cascade and feedback between upper and lower computers [22]. The upper computer is a full-touch tablet PC under Windows XP system with a resolution of 800∗600. The familiar window operating system makes it easy for users to master the operation, while the large high-resolution screen also enhances the user experience. The lower computer is a motor drive system based on ATmega16 chip [23, 24]. The user input the control (button or voice) signal of nursing bed action through the upper computer, and the lower computer is responsible for driving the corresponding motor to perform the corresponding nursing bed action. At the same time, the lower computer detects the limit signal of the relevant position sensor, motor pulse, and voice recognition trigger signal in real time and feeds these signals back to the upper computer for relevant processing. The control system block diagram of nursing bed is shown in Figure 5.

Retrospective analysis was conducted in this study, and 100 subjects were selected, including 50 in the control group and 50 in the intervention group. By comparing the age composition, gender, education level, marital status, per capita monthly income (yuan), payment method of medical expenses, nature of work, and residence of patients in the two groups, the results show that there were no significant differences in age composition, gender, education level, marital status, per capita monthly income (yuan), payment method of medical expenses, nature of work, and residence between the two groups (*P* > 0.05), indicating that the two groups were comparable. In this study, the patients' lumbar function was scored based on the postoperative JOA lumbar function score. Cronbach's A coefficient of this scale was 0.89, which had high reliability and validity. The results showed that there was no significant difference in the JOA lumbar function score between the control group and the day control group (*P* > 0.05). The JOA lumbar spine function scores of the affected group at 1 month and 3 months after operation were 21.2 + 1.010 and 28.34 + 0.939, respectively, which were higher than those of the control group (20.74 + 1.046 and 27.56 + 0.951, respectively). There was significant difference between the two groups (*P* < 0.05). Repeated measure anOVA showed that lumbar function was restored at 1 and 3 months after surgery in both groups over time. However, the recovery of lumbar function in the intervention group was better than that in the control group (*P* < 0.05) [25]. It indicates that the implementation of preoperative lumbar function training guidance, early postoperative exercise, and timely psychological intervention in clinical nursing pathway under ERAS concept can promote the recovery of patients' lumbar function more quickly. It has also been confirmed that ERAS has positive significance for postoperative functional recovery and postoperative pain recovery of patients after knee surgery. ERAS as a concept has been recognized and widely used by medical professionals. The control group was given routine care, while the intervention group was given ERAS care. ERAS care covers multiple aspects of preoperative, intraoperative, and postoperative care, which can reduce the occurrence and duration of postoperative lumbar pain and achieve rapid recovery. Fifteen patients were enrolled in the ERAS observation group. Preoperative drug diagnosis and minimally invasive surgery should be taken to reduce tissue stimulation and dissection in the wound. Postoperative combined analgesic drugs, early functional exercise, reasonable diet, and other methods were used to evaluate the therapeutic effect using VAS. The results showed that VAS score of the observation group was significantly different from that of the control group 1 day after surgery, 3 days after surgery, and at discharge follow-up, *P* < 0.05; ERAS is considered to be an advanced rehabilitation guidance strategy based on evidence-based medicine research, which optimizes management measures for the entire treatment process and every link to embody humanistic care, better communication, and cooperation between patients and medical staff. Early postoperative rehabilitation exercise enhances patient confidence, reduces back pain, prevents nerve root adhesion, and has a good effect [26]. ERAS-assisted modeling has also been shown to improve postoperative pain in perioperative patients. The results of this study showed that there was no significant difference in the VAS scores of the two groups in the days of enrollment (*P* > 0.05). The VAS scores of the patient group on the 1st, 2nd, and 3rd days after operation were 3.38 ± 1.008, 2.30 ± 0.931, and 1.48 ± 0.677, respectively. The lower the control group (4.12 ± 1.466, 2.74 ± 1.225, and 1.88 ± 0.872), the difference was significant, *P* < 0.05. For time (*P* < 0.05), compared with the control group, the pain relief in the affected group was significantly better than the control group (*P* < 0.05). This indicates that during the implementation of clinical nursing pathway under ERAS philosophy for patients, the medical staff has optimized management measures for every link. Timely psychological support for patients, teaching patients to relieve pain methods, enhancing patient confidence, and advancing analgesia and the implementation of multimode analgesia effectively reduce the pain of patients, to achieve the purpose of rapid recovery. Cerebrospinal fluid leakage caused by dura injury is a common complication of lumbar spine surgery. It has been reported that the incidence of cerebrospinal fluid leakage in primary lumbar surgery is 5.5%-9%. Cerebrospinal fluid leakage can cause direct consequences including wound sensation and wound healing, and long time without improvement can cause headache symptoms. The main cause of cerebrospinal fluid leakage is adhesion of ossification and dura, careless operation during the operation, and damage of dura and arachnoid membrane. Prevention is the key to avoid cerebrospinal fluid leakage. Therefore, surgeons must first be familiar with local anatomy, and fully evaluate the adhesion degree between the compressor and the dura, whether there is dura ossification, and fully expose the surgical field during the operation, so as to avoid cerebrospinal fluid leakage as much as possible by improving surgical techniques. For the occurrence of cerebrospinal fluid leakage, actively take the correct treatment method, and strive to achieve good results. The results of this study showed that the incidence of postoperative cerebrospinal fluid leakage was 2% (1 case) in the intervention group and 2% (1 case) in the control group, and there was no statistical significance between the two groups (*P* > 0.05). This may be related to the small sample size of this study, and a large number of clinical trials are still needed in the future to verify the significance of the implementation of clinical nursing pathway under ERAS concept in reducing the incidence of cerebrospinal fluid leakage after lumbar interbody fusion fixation. Urinary retention is a common complication after lumbar surgery. Some studies have found that the incidence of urinary retention after lumbar surgery is 15%. At the same time, patients with lumbar spinal stenosis are prone to urinary tract infection due to routine indwelling catheter after general anesthesia. Foreign studies have reported that the incidence of urinary tract infection after scoliosis and kyphosis surgery is 3.9% and 4.8/%, respectively. The study found that 10.5% of patients developed urinary tract infections after spinal surgery. The incidence of postoperative urinary tract infection varies depending on the population, study, and surgical approach, and patients may experience severe recurrence of postoperative urinary tract infection. Therefore, great attention should be paid to actively intervene to minimize the occurrence of urination and urination [27, 28]. The results of this study showed that the incidence of urinary incontinence and voiding was 4% (2 cases) in the study group and 18% (9 cases) in the study group. The incidence of urinary incontinence and urinary incontinence in the control group was lower than that in the control group, and the difference between the two groups was significant (*P* < 0.05). Li et al. showed that by using therapy in an ERAS strategy, caregivers could reduce urination and urination by educating patients about timely preoperative and appropriate interventions and timely handling of catheters during and after surgery. It is of great significance to prevent urinary retention and urinary tract infection after lumbar interbody fusion and fixation. Abdominal distention often occurs 1~3 days after lumbar spine surgery, which seriously affects the patient's health and mood, diet, and sleep, and increases the patient's pain. Long-term abdominal distention may lead to intestinal adhesion and intestinal obstruction. Abdominal distention may squeeze both lungs and cause dyspnea and dyspnea, which requires extensive attention. Relevant studies on the effects of ERAS on abdominal distention after lumbar spine surgery showed that the incidence of abdominal distension in the observation group (using ERAS nursing) and the control group (using routine nursing) was 7% and 21%, respectively, and the abdominal distension was completely relieved in the observation group 7 days after surgery, while the rate of abdominal distension in the control group was 5%. The difference between the two groups was statistically significant. It is believed that nursing measures under the guidance of BRAS concept can reduce the occurrence of postoperative abdominal distension and relieve abdominal distension as soon as possible, which has great promotion significance. Studies have found that the incidence of postoperative abdominal distension can be significantly reduced through early postoperative activities and functional exercises for patients with lumbar degenerative diseases. In this study, the incidence of postoperative abdominal distension was compared between the two groups. The results showed that the incidence of postoperative abdominal distension was 14% (7 cases) in the intervention group and 32% (16 cases) in the control group, and the difference between the two groups was statistically significant (*P* < 0.05). The results of this study are consistent with the studies of experts outside China, suggesting that the incidence of abdominal distention can be reduced by implementing relevant measures of clinical nursing pathway under ERAS concept, such as fasting for 6 h and 2 h before surgery, small amount of water intake early after surgery, and early ambulation. Deep vein thrombosis of lower limbs is a common complication after orthopedic surgery, which is usually caused by longer operation time, longer postoperative bed time, advanced age, fear of wound pain, and poor postoperative functional exercise. The patient has no obvious symptoms in the early stage, but if not handled in time, the severe case may lead to embolus shedding and pulmonary embolism, endangering the patient's life. Foreign literature has reported that the incidence of venous thrombosis in lower limbs after spinal surgery is 0.3%-31%, and the incidence of deep venous thrombosis in lower limbs in patients with spinal trauma and spinal surgery is 1.2%-3.6%, among which 50%-70% can be secondary to pulmonary embolism. The results vary depending on the population and methods studied. The results of this study showed that the incidence of postoperative deep vein thrombosis in the lower extremity was 0% (0 cases) in the patient group and 2% (1 case) in the control group. There was no significant difference in any one group (*P* > 0.05). There was 1 case of lower extremity deep vein thrombosis in the control group and no case of lower extremity deep vein thrombosis in the intervention group, which was less in both groups. Firstly, it may be closely related to the high attention paid by medical staff, and secondly, it may be related to the small sample size of the study, which still needs to be confirmed by studies with large samples in the future. Wound infection can be seen in a variety of factors. Studies have found that the causes of wound infection after lumbar interbody fusion fixation are often diabetes, infection history, long operation time, smoking, and interbody fusion device implantation. Previous back surgery and diabetes were reported to be significant risk factors for wound infection. It has been reported that the incidence of incisions after lumbar spinal stenosis is 4% to 6%, and the incidence of incisions after lumbar spinal stenosis and interbody fusion is 2.5%. The results of this study showed that the incidence of postoperative pain in the intervention group was 2% (1 case), and that in the control group was 10% (5 cases), with no value in either group (*P* > 0.05). This may be related to the small sample size of this study and the improvement of medical asepsis technology. Future studies with large samples are still needed to confirm the significance of clinical nursing pathway implementation under ERAS concept in preventing wound infection after lumbar interbody fusion fixation.

## 5. Conclusion

Here, a BTS (brain tumor) operation training simulator was developed from the training of neurosurgery, aiming to solve the practical problems of difficult training and high cost in neurosurgery. And the existing problems in virtual neurosurgery are introduced, and the key problems in virtual neurosurgery are studied. The basic training module of BTS surgery was designed, and the simulator was analyzed subjectively and objectively to verify its effectiveness. The main work of this essay includes the following aspects: surface rendering and volume rendering in 3D reconstruction of medical images are compared, and volume rendering of medical images based on Ray Casting algorithm is realized in Unity3D, which plays a crucial role in preoperative planning of virtual surgical simulator. The soft tissue modeling and cutting in neurosurgery were realized based on XPBD algorithm, and surgical training modules such as skin cutting were realized in Unity3D, which further improved the simulator of brain tumor surgery. A grid voxel method was proposed to reconstruct the skull, and a training module for craniotomy was designed to solve the problem of unreal tactile simulation in orthopedic surgery.

## Figures and Tables

**Figure 1:** Flow chart of neurological examination under microscope.

**Figure 2:** The relationship between attractiveness and belonging.

**Figure 3:** Pie chart of satisfaction score of intervention group.

**Figure 4:** Overall framework of nursing bed experimental platform.

**Figure 5:** Control system block diagram of nursing bed.

**Table 1:** Comparison of nursing satisfaction score between intervention group and control group (*n*(%)).

	Quite satisfied	Satisfied	So-so	Dissatisfied	*Z* value	*P* value
Intervention group (*n* = 50)	7 (14)	31 (62)	10 (20)	2 (4)	-3.208	0.001
The control group (*n* = 50)	4 (8)	15 (30)	26 (52)	5 (10)		

**Table 2:** Basic monomer movements of nursing bed.

Left side	Left turn up	Right side	Right turn up
	Left turn down		Right turn down

North	Back up	Legs	The leg up
	Back down		The leg down

The head of a bed	Bed body rise	The end of the bed	Bed rise
	Bed body down		Bed down

## Data Availability

The data used to support the findings of this study are available from the corresponding author upon request.
